The article "The Effects of Different Reference Methods on Decision-Making Implications of Auditory Brainstem Response" was published in 2022. Journal: Comput Math Methods Med.

# The Effects of Different Reference Methods on Decision-Making Implications of Auditory Brainstem Response

**DOI:** 10.1155/2022/9923214

**Published:** 2022-04-08

**Authors:** Zhenzhen Liu, Xin Wang, Mingxing Zhu, Yuchao He, Lin Li, Li Chen, Weimin Huang, Zhilong Wei, Shixiong Chen, Yan Chen, Guanglin Li

**Affiliations:** ^1^Surgery Division, Epilepsy Center, Shenzhen Children's Hospital, Shenzhen 518038, China; ^2^The CAS Key Laboratory of Human-Machine Intelligence-Synergy Systems, Shenzhen Institutes of Advanced Technology, Chinese Academy of Sciences, Shenzhen 518055, China; ^3^Shenzhen College of Advanced Technology, University of Chinese Academy of Sciences, Shenzhen 518055, China; ^4^Guangdong-Hong Kong-Macao Joint Laboratory of Human-Machine Intelligence-Synergy Systems, Chinese Academy of Sciences, Shenzhen 518055, China; ^5^Department of Neurology, Shenzhen Children's Hospital, Shenzhen 518038, China; ^6^Department of Neonatology, Shenzhen Children's Hospital, Shenzhen 518038, China

## Abstract

Hearing loss is a common disease affecting public health all around the world. In clinic, auditory brainstem response (ABR) has been widely used for the detection of hearing loss based on its convenience and accuracy. The different reference methods directly influence the quality of the ABR waveform which in turn affects the ABR-based diagnosis. Therefore, in this study, a reference electrode standardization technique (REST) was adopted to systematically investigate and evaluate the effect of different reference methods on the quality of ABR waveform in comparison with the conventional average reference (AR) and mean mastoid (MM) methods. In this study, ABR signals induced by click stimulus were acquired via an EEG electrode cap arrays, and those located on the six channels along the midline were compared systemically. The results showed that, when considering the different channels, the ABR in the Cz channel showed the best morphology. Then, the ABR waveforms acquired via the REST method possessed better morphologies with large amplitude (0.06 ± 0.02 *μ*V for wave I, 0.07 ± 0.02 *μ*V for wave III, and 0.21 ± 0.04 *μ*V for wave V) when compared with the traditional method. Summarily, we found that the REST and MM methods improved the quality of ABR on both amplitude and morphology under different stimulation rates and levels without changing the latencies of ABR when compared with the conventional AR method, suggesting that the REST and MM methods have the potential to help physicians with high accurate ABR-based clinical diagnosis. Moreover, this study might also provide a theoretic basis of reference methods on the acquisition of electroencephalogram over public health issues.

## 1. Introduction

Hearing loss has been reported to affect over 1.1 billion individuals across different age groups, which causes a huge public health issue. In clinical settings, auditory brainstem response (ABR) has a decision-making implication on hearing loss diagnosis based on its accuracy, convenience, and efficiency. ABR was firstly described in detail by Jewett et al. in 1971 as a potential change in the auditory nerve pathway from the cochlea to the brainstem evoked by an acoustic stimulus and could be recorded noninvasively on the scalp of the subjects [1]. As a matter of fact, ABR is the most commonly applied auditory-evoked responses in clinical settings because it allows adequate assessment of the auditory neural pathway and hearing sensitivity [2, 3]. Fundamentally, ABR is composed of seven waveform peaks, in which the first five are often used for hearing loss assessment in clinical practice. The peaks are classified based on their temporal appearance as described by Jewett and Williston (waves I-V) [4]. Each of the five waves (waves I-V) has been characterized and attributed to different anatomical region in auditory pathway [5]. The indexes used to recognize an ABR waveform are wave latency, interwave latency, waveform repeatability, and so on. The occurrence of abnormality in ABR waveform, like a disappearance of subsequent waves and the change of wave latency, provides a basis for the localization of the auditory nerve and brainstem auditory pathway lesions.

The quality of the ABR waveform is considered as a core determinant for the effective assessment of hearing loss and its associated cause. Many research focus on the improvement of physiological signal's quality by applying deep learning methods [6–10]. Similar as other physiological electrical signals, ABR is a potential difference-based signal that is recorded against a specific reference point. However, ABR signals are mainly characterized by weak amplitudes that typically range between 0.1 and 0.9 *μ*V [11], thereby making it susceptible to interferences resulting from the electrical activity of the reference electrode. In electroencephalogram (EEG) studies, the commonly employed reference electrode methods include vertex (Cz), mean mastoid (MM), and average reference (AR) approaches [12]. Characterized by various advantages, each method also has some limitations in some ways. For instance, when the Cz reference approach is utilized, the recorded signals are usually affected by the electrophysiological activities around the Cz point [13]. For the MM approach, the average of the two mastoid electrodes is subtracted from the potential per time, which is a function of the potential changes associated with the mastoid electrodes [14]. Meanwhile, for the AR approach, the recorded data per electrode is subtracted from the overall average across electrodes per time, which is the most commonly adopted scheme, especially in the context of multichannel EEG signal analysis [15, 16]. Despite its wide adoption, the AR approach is characterized by some issues that have limited its adoption in large-scale clinical and commercial settings. One of such critical issues is that the potentials evoked based on the AR method do not only depend on the changes in the reference point but also on the potential changes that occur in the other surrounding electrodes. Besides, in situations where the selected reference points are different from absolute zero potentials, the ABR signals become inevitably affected.

In selecting a reference electrode, the potential should be as close to zero as possible; however, such point rarely exists on the scalp [17]. Meanwhile, inevitable alterations in the voltages at the reference electrode will cause a change in the recorded potential of the active electrode [18]. Therefore, in situations where the reference electrodes are different, the waveforms recorded from the same active electrode position would vary largely leading to inconsistent results [19]. In other words, the choice of the reference electrode is a key issue in obtaining reliable evoked potentials during EEG signal acquisition. In order to minimize the impact of reference electrode on evoked potential detection, previous studies have proposed the use of different kinds of reference methods [20–24]. For instance, in 2001, Yao proposed a “reference electrode standardization technique (REST)” that could approximately convert brain response recordings with a point on the scalp and an average potential as a reference with respect to a spatial infinity point [25]. The physical basis of the method is that the potentials before and after the conversion are generated by real neural activity in the brain or its equivalent distribution, such that the potentials before and after the conversion can be linked by a common physical source [26]. Yao et al. also proved the effectiveness of their proposed REST in the context of EEG spectral mapping [27], EEG default mode networks [28], and other event-related potentials (ERPs) [29–31].

To date, to the best of our knowledge, the application of REST in ABR for an effective assessment of hearing loss has not been conducted. Therefore, as a crucial step towards the effective evaluation of hearing loss, we systematically investigated the possibility of adopting REST technique for qualitative ABR signal assessment and subsequently compared its effectiveness with the commonly applied conventional AR and MM reference methods. Furthermore, we examined the influence of different reference methods on the quality of the acquired ABR waveforms with respect to the AR, REST, and MM methods while considering different stimulus rates and test levels. Meanwhile, we utilized 30 channels from a 64-channel EEG acquisition system to record ABR signals and compared the ABR waveforms at midline positions, especially the Cz channel. Finally, we studied the differentiable characteristics of the ABR waveforms across the three examined methods especially considering waves I-III-V and their amplitude properties to ascertain their merits and demerits with respect to hearing loss assessment. Finally, we studied the characteristics of ABR across the three examined methods by considering those typical wave (I, III, and V) morphologies and their amplitudes to ascertain their merits and demerits on hearing loss assessment.

## 2. Methods

### 2.1. Participants

In this study, a total of ten subjects without hearing defect (6 males and 4 females) with age range between 20 and 28 years (mean age = 24.6 years) were recruited for the EEG data collection. Prior to the experimental design, a standard audiogram test was carried out, and those whose audiogram thresholds were 20 dB hearing level (HL) or less for frequencies between 250 and 8000 Hz were chosen. The participants were properly briefed about the aim of the study and details of the experiments; afterward, a consent form indicating their willingness to participate in the study was signed by all the subjects. The entire experimental protocols were approved by the Institutional Review Board (IRB) of the Shenzhen Institutes of Advanced Technology, Chinese Academy of Sciences (SIAT-IRB-180415-H0252).

### 2.2. Equipment and Setup

The EEG recordings used to extract the evoked ABR signals were recorded using a Neuroscan SynAmps^2^ (*NeuroScan, Inc.*) acquisition system. In the amplifier settings section, the sampling rate was configured to 20000 Hz and AC mode was selected. Then, the low pass filter was set to 3000 Hz, while the high pass filter was configured with a cut-off frequency of 100 Hz. Afterwards, the corresponding ABR signals were recorded using Ag/Agcl with 64-channel Quik-cap (*Neuromedical Supplies, Sterling, USA*), and according to the international extended 10/20 montage, 32 channels out of the 64 channels were considered for the analysis in the study [32]. Meanwhile, 30 channels out of the 32 channels are presented in Figure 1(a), and these channels are FP1, FP2, F7, F3,Fz, F4,F8,FT7,FC3,FCz, FC4, FT8, T7, C3, Cz,C4, T8, TP7,CP3, CPz, CP4, TP8,P7, P3, Pz, P4, P8, O1, Oz, and O2. Among these electrode channels, Fz, FCz, Cz, CPz, Pz, and Oz channels were arranged along the midline of the skull, while the remaining electrodes were located symmetrically on both sides of the midline (Figure 1(a)). Besides, the GND and REF electrodes on the EEG cap served as ground and online references, respectively. The remaining two channels were placed on the left and right mastoids (M1 and M2), which were later used for rereference purpose. For reconstructing the head model, a three-dimensional (3D) digitizer (*Polhemus, Colchester, VT, USA*) was used to measure the EEG electrodes' location on the scalp. As shown in Figure 1(b), the receivers of the 3D digitizer are placed on the left and right temples and occipital bulge, forming a triangular plane. The transmitter is placed on a tripod that is about 30 cm away from the subject's face, while the *x*-axis is positively oriented towards the subject's face. Sequentially, the selected electrodes were located according to the amplifier setting file.

### 2.3. Stimuli and Procedures

Generally, click-induced ABR method has been considered as a benchmark approach for estimating hearing loss [33]; hence, it was utilized as the stimulus mechanism produced by a customized printed circuit board (PCB) controlled by a MATLAB program in this study. Basically, click is referred to as a broadband signal, which is generated by an electric pulse with a width of 100 *μ*s into the earphone. It should be noted that during the experiment, the stimuli were presented to the subject's left ear by an ER-2 insert earphone (*Etymotic Research Inc.*), with an earplug in the right ear. Besides, the stimuli were calibrated in normal hearing level (nHL) with an occluded ear simulator. Click-evoked ABRs that employed AR, REST, and MM reference methods were compared at different stimulus rates and levels.

Prior to the experiments, the participants were required to properly clean their hair so as to minimize the impedance between the electrodes of the Quik-cap and their scalp. Afterwards, they were told to sit in a comfortable chair in an acoustically and electromagnetically shielded room in a relatively calm/quiet manner. The Quik-cap was worn on the subject's head, and all the electrode impedances were maintained below 5 k*Ω*. Before the ABR acquisition commenced, the locations of the selected electrodes on the scalp were measured by the abovementioned 3D digitizer, and the 3D coordinates of the electrodes were captured and stored for further processing.

In the experiment, the ABR signal acquisition was accomplished in two sessions. In the first experimental session, we considered various stimulus rates including 10/s, 25/s, 50/s, and 100/s, in which the stimulus level was set at 75 dB nHL. Meanwhile, in the second experimental session, a constant stimulus rate of 25/s was applied, while the stimulus level was varied between 45 and 80 dB nHL, with the interval of 5 dB nHL. Meanwhile, each trial consisted of 4000 averages, and two independent trials were recorded for each stimulus condition to verify the repeatability of the response. It should be noted that the subjects were allowed to rest for about five minutes after every four trials to avoid nervous system-inclined fatigue which may affect the quality of the ABR recordings. Thereafter, the experiments for each subject lasted for about two hours, and the raw recorded data were saved on a storage device for subsequent offline processing and analysis.

### 2.4. Data Analysis

The acquired data were analyzed using the EEGLAB toolbox [34] that was integrated into MATLAB (*MathWorks Inc., USA*) computing software environment. The raw signals were firstly preprocessed by applying a 3 order butter worth band pass filter with cut-off frequencies of 100~1500 Hz. To investigate the effects of different reference electrode configurations on the signals' characteristics, the preprocessed EEG data (recorded via Ref as reference electrode) was reconstructed offline based on the AR, MM, and REST methods, respectively (Figure 2).

The AR and MM methods were implemented via the *pop_reref* inbuilt function in EEGLAB toolbox. In principle, the AR reference method could be realized by computing the average of all channels, while the MM method could be achieved by averaging the signals obtained from the left and right mastoids (also known as the average of the data from the M1 and M2 channels). Further, the REST method was implemented by converting the reconstructed signals via the REST EEGLAB plugin module developed by a group of researchers from the University of Electronic Science and Technology, Chengdu, China [25].The reconstruction process, which was shown in Figure 3, based on the REST module actually began with the execution of a program file named the *LeadField.exe* that firstly converted the 3D coordinates of the previously acquired signals to obtain a transfer matrix. Then, the EEG signal and the transfer matrix were converted to the REST-referenced data by utilizing *pop_REST_reref* inbuilt function. Thereafter, the EEG data reconstructed based on the three reference methods (AR, MM, and REST) were exported to the MATLAB programming environment for further analysis. It was worth noting that the continuous EEG data were divided into epochs with 10 msat the onset of each stimulus. Because the ABR is a low-amplitude signal and auditory-evoked potential, the ABR was extracted from the noised EEG signals by averaging technique to average all the segmentations. In this study, the target ABR signals were obtained by averaging 4000 epochs.

After a successful reconstruction process which took around 10 minutes, the effects of the different reference methods on the ABR waveform characteristics were examined by comparing the waveforms of the following electrode locations: Fz, FCz, Cz, CPz, Pz, and Oz in the midline using AR and REST reference methods. In addition, we compared the waveforms of the Cz channel when the reference methods were the AR, MM, and REST, focusing on the extent of waveform differentiation and wave V latency of ABR in the Cz channel with the stimulus rate and level.

## 3. Results

### 3.1. Analysis of ABRs Obtained along the Midline Channels via the AR and REST Methods

In this analysis, the ABR signals obtained via the AR and REST methods from the electrodes placed along the midline channels on the Quik-cap were analyzed and compared. From the processed data, it was observed that the signals picked up by the electrodes at the midline were better than those at other locations on the scalp. Therefore, we considered the ABR waveforms on Fz, FCz, Cz, CPz, Pz, and Oz electrodes located on the midline of the scalp in our subsequent analysis. As shown in Figure 4, a comparative analysis of the ABR waveforms obtained via the AR and REST methods from the abovementioned electrode channels at 75 dB nHL with a rate of 10/s was carried out. From the results, waves I, III, and V of ABR obtained from AR and REST on the Fz, FCz, Cz, CPz, and Pz channels could be clearly identified, while the ABR waveform processed by the REST method was observed to have a larger amplitude compared to that of the AR method. Moreover, the ABR waveform constructed from the Oz channel located on the occipital region using the AR method is poorly differentiated, thereby making it relatively difficult to identify the peaks in waves I, III, and V. Meanwhile, the ABR signals recorded at the Oz channel via the REST method were seen to be better than those obtained via the AR method, with clearly distinct wave V. In summary, regardless of the selected channel, the quality of the ABR waveform obtained via the REST method was observed to be better than that obtained from the AR method. Furthermore, we discovered that the ABR waveforms' differentiation in the Cz channel appeared to be the best irrespective of whether the AR or REST method was adopted for obtaining the ABR recordings. Hence, we considered the ABR recordings obtained from the Cz electrode channel in our subsequent analysis.

### 3.2. Comparison of ABR Signals in the Cz Channel Using the AR, REST, and MM Methods

In view of the above findings, we selected and compared the responses of the Cz channel recorded via the AR, REST, and MM methods under the condition of 75 dB nHL and 25/s (Figure 4). By carefully observing the waveforms in Figure 5, it could be seen that the amplitude of the ABR signals obtained via the AR method was slightly lower (only 0.1 *μ*V) compared to that of the other two methods. Although the waves I-V could be adequately recognized, their differentiation seemed to be poor, especially those of waves IV and V. Compared with the AR method, the ABR waveform obtained via the REST method has better differentiation and higher amplitude characteristics, while the waveform differentiation of the ABR recordings obtained via the MM method was similar to that of REST but with relatively higher amplitudes. Although the amplitude of ABR signals was different with different reference methods, the latency of ABR waves I-V obtained was the same.

Table 1 shows the mean amplitudes and the standard deviation of waves I, III and V for ABRs obtained by the AR, REST, and MM methods across all the subjects (*N* = 10 ears). Obviously, the ABR obtained by the MM method had the highest mean amplitudes, and its wave V mean amplitude was as high as 0.27 *μ*V. The mean amplitudes of the ABR obtained via the REST method were lower than those of the MM method, in which the mean amplitude of wave V was 0.21 *μ*V. The mean amplitude of the ABR by the AR method was the lowest, with the mean amplitude of wave V of 0.08 *μ*V.  Table 2 showed the mean and standard deviation of interwave latencies for waves I-III and III-V of ABRs obtained by the AR, REST, and MM methods, which were derived from the same raw data as Table 1. As shown in Table 2, the ABRs obtained by the three reference methods (AR, REST, and MM) had the same interwave latencies for waves I-III and III-V, which proved that the reference methods could improve the ABR on the aspect of amplitude but without essentially affecting the waveform on the latency.

### 3.3. ABRs of the Three Reference Methods in the Cz with Different Stimulus Rate and Intensity

To further examine whether the conclusion reached in the previous analyses (Figure 4) could be influenced by variation in stimulus rates and levels, we compared the ABR waveforms of the Cz channel using the AR, REST, and MM methods under the influence of varying stimulus rates and levels, and the experimental results were presented in Figures 6 and 7.  Figure 6 represented the ABR waveforms obtained using the Cz channel at a stimulus level of 75 dB nHL under stimulus rates of 10/s, 25/s, 50/s, and 100/s. It could be noticed in Figure 6 that the latency of wave V increased with a corresponding increase in stimulus rate, while the waveform at lower stimulus rate was observed to have better waveform differentiation characteristics (waves I-V). These findings were in line with the conclusion of a previous study [35], and we also found that a correlation existed between the latency and stimulus rate regardless of the reference method adopted. This invariably meant that regardless of the stimulus rate (10/s, 20/s or 50/s) applied, the five peaks (waves I-V) of the ABR waveform obtained via the AR method would still be inadequately differentiated. Meanwhile, the waveforms of the ABR obtained via the REST and MM methods at the stimulus rates of 10/s, 20/s, and 50/s, were well differentiated, especially when the stimulus rate was set to 10/s (Figure 6). This phenomenon exhibited by the examined reference methods would result in easy recognition of the ABR waveforms in the context of the five peaks (waves I-V). Furthermore, the amplitudes of the ABR signals obtained through the REST and MM methods were obviously higher than those of the AR method. When considering the ABR under stimulus rate of 100/s, the waveforms obtained via the three reference methods become less distinguishable, which might be due to the stimulus interval of only 10 ms, resulting from the middle latency component of the response induced by the previous stimulus affecting the ABR induced by the latter stimulus. Compared with the ABR obtained via the AR method at the rate of 100/s, waves III and V could also be clearly identified using the REST and MM methods.

From Figure 7, it could be observed that the ABR recordings of the Cz channel obtained via the three reference methods at a rate of 25/s exhibited different characteristics. Moreover, the ABR latency was delayed, and the waveform differentiation became worse with a decrease in stimulus intensity. It should be noted that these trends were independent of the reference methods. Therefore, regardless of the stimulus level, the ABR waveform differentiation obtained via the AR method was not as good as the ones obtained through the REST and MM methods. Meanwhile, at the same stimulus level, the MM method had the largest amplitude followed by the REST method, and the AR method was with the smallest ABR amplitude. It should be noted that this phenomenon was consistent with the conclusion drawn from Figure 5.

## 4. Discussion

The main contribution of this study was to investigate the characteristics of the REST technique of ABR signal processing in comparison to the commonly applied reference methods, which helped with the improvement of the ABR-based decision-making implication on hearing loss. Although we utilized the Quik-cap EEG system to acquire 30 channels of ABR signals, only the recordings of 6 channels located along the midline were considered for the study, based on the analysis of the signal quality. Specifically, we compared the ABR signals corresponding to the Cz channel obtained via the AR, REST, and MM methods and their characteristics when subjected to different stimulus rates and levels. From series of experimental results, we found that the REST method would be effective for ABR signal recording, and the quality of the ABR signal obtained via the REST technique was much better than that of the conventional AR method, but not superior to that of the MM method. In addition, a similar phenomenon for the three methods was observed across different stimulus rates as well as levels.

### 4.1. ABRs in the Midline Channels via the AR and REST Methods

In order to verify the feasibility of applying the REST method for ABR signal acquisition, we compared the ABR recordings obtained by the REST method with that obtained via the traditionally applied AR method. Preliminary processing of the raw data showed that the quality of ABR waveforms obtained from the midline channels was better than that of the other channels. Besides, the electrodes located at the vertex or forehead were usually chosen as the active electrode in the single-channel ABR acquisition [36]. Similar to the findings of this study, Moulton et al. proposed a midline electrode configuration that could avoid priority recording from either side of a subjects' head [37]. In line with these previous studies, we compared the ABR signals of the six channels (Fz, FCz, Cz, CPz, Pz, and Oz) along with the midline position as shown in Figure 3, and the experimental results showed that the ABR waveforms obtained via the REST method were obviously distinguishable compared to those of the AR method, which was also consistent with the findings on event-related potential by Dong et al. [38]. It should be noted that the AR method was based on the average potential of all recording electrodes, which was affected by the density of the electrodes. Theoretically, when the scalp electrodes are dense enough, the potential obtained via the AR method would approach the expected value [39]. Thus, the REST method can approximately correct the reference value to the infinite point and therefore make up for the disadvantage that the conventional method has.

### 4.2. ABRs in Cz Channel Obtained via AR, REST, and MM Methods

From Figure 3, the ABR signal at the Cz channel appeared to provide best performance among the electrodes on the midline, which was consistent with the findings from the previous studies on auditory-evoked potentials [40, 41]. In this direction, Beattie and Lipp compared the latency and amplitude of the ABR collected from the vertex and the forehead as active electrodes, respectively [40]. Their results showed that there was no significant difference in the latency and interwave latency between the two active electrode positions, but the wave V amplitude of the ABR obtained from the vertex was larger than the one obtained from the forehead. Therefore, the ABR waveform of the Cz channel was mainly focused and compared as presented in Figure 4. Meanwhile, the results indicated that the amplitude of the ABR waveform obtained through the MM method was the highest, followed by the REST method, while the AR method was the smallest. This conclusion was consistent with the findings from a previous study on auditory mismatch negativity by Mahajan et al. [42]. Hence, we concluded that the ABR amplitude obtained via the MM method was larger than that of REST, which may be due to the fact that bilateral mastoids are adjacent to the ankle occipital region, where task-related electrical activities are inevitably incorporated into the calculation of MM reference method. In most cases, this weakens the signal in the bilateral occipital region, while the amplitude of the signal away from the bilateral mastoid site (i.e., the central frontal region) may increase erroneously. The potential error at the mastoid may also increase the amplitude of the Cz channel, resulting in a larger amplitude of ABR for the MM method than for the REST method.

### 4.3. Characteristics of the ABRs Obtained across Stimulus Rates and Levels

The morphology of the ABR waveforms obtained via the REST and MM methods was obviously better than that obtained via the AR method. When the stimulus condition was set at 75 dB nHL and a rate of 25/s, the ABR amplitude of the MM method appeared to be the largest, followed by the REST method, and the AR method ranked last, which was verified in Figure 4. Meanwhile, Figures 5 and 6 presented the comparative results of ABR obtained by the three reference methods with adjustments in stimulus rates and levels. Regardless of what stimulus rates and levels were applied, the ABR obtained via the MM and REST methods was often better than the AR method. This invariably meant that the conclusions from Figure 4 were valid. However, the latency of the ABR obtained based on the three reference methods was always the same, even if the stimulus rate and level change. This meant that the reference method only changes the representation of the ABR signal, without affecting the nature of the signal, since the physician always make the diagnosis based on the characteristics of the latency. This clearly demonstrated that an effective reference method could efficiently reconstruct the target signal towards improving its quality.

In addition, the latency of the ABR waveform was observed to be highly prolonged with a corresponding increase in the stimulus rate. Moreover, the lower the stimulus rate, the better the waveform differentiation of waves I-V. However, when the stimulus rate was much high, for instance, 100/s, the ABR obtained through the three reference methods becomes very poor (Figure 5). This is possible for the following reasons. The ABR is an early component of auditory-evoked potential (AEP), which occurs between 0 and 10 ms after an acoustic stimulus, and it is characterized by an auditory middle latency response (MLR) after the acoustic stimulus 10 ms [43]. When the stimulus rate is 100/s, the stimulus interval is only 10 ms, which results in the MLR induced by the previous stimulus superimposed on the ABR waveform induced by the latter stimulus. Therefore, whether reference methods are applied, it is necessary to keep the stimulus rate lower than 100/s to assure a meaningful ABR can be acquired.

### 4.4. REST for Medical ABR Application Scenarios

In clinical, the physicians make diagnosis based on the characteristics of ABR such as the morphology, the amplitude of waves, the wave latency, and the interwave latency [44, 45]. However, all these parameters needed are heavily related to the ABR signal quality and the morphology. For example, the interwave latency of waves III and IV could be used to infer the axonal conduction time, while the interwave latency of IV and V represents a synaptic delay [46]. Besides, as reported by J. Lee et al., the amplitude of wave II was regarded as an indicator that helped in diagnosing vestibular paroxysmia [47].Therefore, once the ABR quality or morphology is poor, the parameters needed will be obscure which will also cause difficulty for the physicians to make corresponding diagnosis. Hence, it is meaningful and helpful to improve the ABR quality on the aspects of morphology and amplitude. In this manuscript, the REST-based ABR had been systematically investigated in comparison with the traditional AR method. Our results suggested that the REST method could significantly improve the amplitude of waves I (0.06 ± 0.02 *μ*V), III (0.07 ± 0.02 *μ*V), and V (0.21 ± 0.04 *μ*V) when compared with the traditional AR methods (0.02 ± 0.02 *μ*V for wave I, 0.03 ± 0.01 *μ*V for wave III, and 0.08 ± 0.03 *μ*V for wave V). Moreover, it should be pointed out that the improvement on the morphology and amplitude of ABR was achieved by unchanging the latency of each wave, which meant that the REST method-based ABR could provide physicians as the consistent latency-based information as the traditional AR method did. In consequence, the REST method would assist physicians in ABR-based diagnosis of hearing loss and other auditory diseases, with the significant improvement in ABR morphologies, making it more meaningful in medical application scenarios.

## 5. Conclusions

The study demonstrated that the REST method could be effectively applied for high-quality ABR signal recording, which might be potential for the improvement of ABR-based decision-making implications over the public health issue like hearing loss. The ABRs obtained via the MM and REST methods had better waveform morphologies in comparison to that of the AR method. Moreover, the ABR amplitude obtained through the MM method was observed to be the highest, followed by the REST, and subsequently the AR method. In addition, the latency of the ABRs obtained by the AR, REST, and MM methods appeared to be the same under the same stimulus conditions. This phenomenon was also observed across different stimulus rates and levels, which meant that the reference methods only affected the degree of differentiation and amplitude of the ABR waveform, without changing the latency of each peak. For the ABR signals, the amplitude, which was an important indicator in EEG research, would be directly affected by the selected reference method as shown in our experiments. Therefore, the selection of an objective and effective reference method could help improve the quality of the ABR waveform and aid efficient signal analysis and processing that may be potential in clinical applications.

## Figures and Tables

**Figure 1:** Electrode position distribution map and demonstration of 3D location of the electrodes on the scalp of a representative subject. (a) The distribution of the selected electrodes on the scalp of a representative subject according to the 10/20 international system standard. (b) The constructed head model based on the locations of the selected electrodes on the scalp by a 3D digitizer.

**Figure 2:** The schematic diagram of ABR acquisition and processing from raw EEG signals.

**Figure 3:** The flow chart of the given three algorithms.

**Figure 4:** A representation of ABR waveforms of six channels along the midline (Fz, FCz, Cz, CPz, Pz, and Oz) at 75 dB nHL and a rate of 10/s. (a) Top row panels represented ABR obtained via the AR method. (b) Bottom row panels represented ABR obtained via the REST method.

**Figure 5:** Representation of ABR waveforms of the Cz channel using the AR, REST, and MM reference methods under the condition of 75 dB nHL and 25/s.

**Figure 6:** The ABR waveforms of the Cz channel obtained via the AR (left panel), REST (middle panel), and MM (right panel) methods, correspondingly. Note: the stimulation level is 75 dB nHL, and the stimulus rate varies from 10 to 100/s, as indicated.

**Figure 7:** The ABR waveforms of the Cz channel obtained via the AR (left panel), REST (middle panel), and MM (right panel) methods, respectively. The stimulation level varied from 80 to 45 dB nHL, and the stimulus rate was 25/s.

**Table 1:** The amplitudes (*μ*V) of waves I, III and V of the ABRs obtained by the AR, REST, and MM methods at a level of 75 dB nHL and a rate of 25/s (mean and standard deviation; *N* = 10 ears).

Method	Wave I		Wave III		Wave V	
	Mean	SD	Mean	SD	Mean	SD
AR	0.02	0.02	0.03	0.01	0.08	0.03
REST	0.06	0.02	0.07	0.02	0.21	0.04
MM	0.09	0.04	0.11	0.05	0.27	0.07

**Table 2:** The interwave latencies (ms) for waves I-III and III-V of the ABRs obtained by the AR, REST, and MM methods at a level of 75 dB nHL and a rate of 25/s (mean and standard deviation; *N* = 10 ears).

Method	Wave I-III		Wave III-V	
	Mean	SD	Mean	SD
AR	2.05	0.11	1.95	0.08
REST	2.05	0.11	1.95	0.08
MM	2.05	0.11	1.95	0.08

## Data Availability

The data used to support the findings of this study are available from the corresponding author upon request.
